# Evaluation of Tourism Food Safety and Quality with Neural Networks

**DOI:** 10.1155/2022/9493415

**Published:** 2022-08-16

**Authors:** Dandan Li, Shuai Wang, Ang Zhao

**Affiliations:** ^1^Key Laboratory of Food Science and Technology, School of Life Sciences and Food Engineering, Nanchang University, Nanchang 330047, China; ^2^Liyang Culture Sports Radio Film and Tourism Bureau, Liyang 213300, China; ^3^Shandong Polytechnic, Jinan 250104, China; ^4^Minquan County Vocational and Technical Education Center, Minquan 476800, China

## Abstract

Food safety issues are inextricably linked to people's lives and, in extreme cases, endanger public safety and social stability. People are becoming increasingly concerned about food safety issues in a modern society with high-quality economic development. People's incomes are increasing day by day as the economy continues to grow, and the tourism industry has grown by leaps and bounds. However, many problems arose, such as the issue of food safety in tourism. Tourism food safety issues affect not only the development of the food industry but also the development of tourism. Food safety oversight of tourist attractions has always been a relatively concerning issue in the country, and it is also something that the general public is concerned about. It can be said that food safety supervision of tourist attractions is the most important thing in food safety supervision. In this context, it becomes an important task to evaluate the safety of tourist food. This work proposes a multiscale convolutional neural network (AMCNN) combined with neural networks and attention layers to realize the safety and quality evaluation of tourist food. The algorithm uses the lightweight Xception network as a basic model and utilizes multiscale depth-separable convolution modules of different sizes for feature extraction and fusion to extract richer food safety feature information. Furthermore, the convolutional attention module (CBAM) is embedded on the basis of the multiscale convolutional neural network, which makes the network model focus more on discriminative features.

## 1. Introduction

Tourism has become an important part of people's daily lives, and holiday travel has become a very important way of consumption for people to meet their daily needs. China not only has a large population but also is very rich in tourism resources. Tourism includes play, food, accommodation, shopping, and many other aspects and plays an important role in promoting the development of the national economy. Food in tourist attractions is an important part of tourism, and food has always played an important role as an element in the process of tourism. Particularly, now, a lot of tourism activities are themselves food-centric. For example, various food festivals and beer festivals are often held all over the country, and the purpose of tourism is to consume various foods, so the importance of food safety in tourism is obvious. Food safety is a priority for most people. Food safety in tourist attractions not only is related to the health of every tourist but also highlights the image of a region as well as the economic development and social stability of the region. In the tourism income of domestic tourists, the proportion of the main tourism of the six elements of food, accommodation, travel, shopping, and entertainment is not large, and the scenic spot ticket income only accounts for 2.37% of the total tourism income. However, the income from eating, accommodation, transportation, shopping, entertainment, and so on generated by its drive accounted for 97.63%, and food consumption accounted for a large proportion [1–5].

Tourism food safety mainly covers the following points: first, the catering services that tourists receive in restaurants, tourist attractions, and the means of transportation they take; second, buying special food products in tourist attractions and on the way; third, the catering services, food shopping, and picking activities that tourists receive during the travel process that may have food safety problems. Particularly in some tourism products centered on food, such as some food festival tourism and snack square tourism, it is more likely to become the source of food safety problems. First of all, the country has a large population and a large tourist population base. Once a tourist food safety problem occurs, its control and investigation are extremely difficult. Second, consumers are highly mobile, and some specific travel groups may even travel across multiple provinces or even countries or regions along the travel agency's established routes. As a result, food safety incidents can be far away from where they occur and where they are discovered. Then, there is a big difference in the number of tourists in the peak and low seasons of tourism. This results in the neglect of food safety issues due to the increase in the number of receptions during the peak tourist season, thereby increasing the chance of food safety issues. Finally, the economic base of tourist destinations varies widely. Some tourist destinations with poor economic foundations have relatively weak food safety awareness and food safety supervision. At the same time, limited by the local equipment and sanitary conditions, it is difficult to provide a scientific and effective food safety guarantee for tourists [6–10].

The main reasons for the safety and quality of tourism food are as follows. First, the potential food safety crisis in the tourism food industry chain is a complex system, and the links included in the industry chain vary with the type of tourism food. Generally speaking, the main components of the tourism industry chain include six major links: planting (breeding), processing, storage, transportation, sales, and consumption. Any problem in any link will have a negative impact on the health and food safety experience of tourists. Since the tourism food industry chain is long, problems in each link will have an impact on the safety of the final tourism products, further increasing the probability of tourism food safety problems. At the same time, it also increases the difficulty for the regulatory authorities to investigate and supervise food safety incidents. Second is the information asymmetry in the tourism food industry chain. Particularly between tourists and tourist food producers and operators, there is a high degree of information asymmetry. Tourists have little knowledge of local tourist food information after entering a specific tourist area. However, travel agencies and tourist food operators often transmit information on the quality and safety of tourist food through selective filtering from the perspective of their own interests, which misleads tourists' consumption choices to a certain extent. Third, the scale of the tourism food industry chain is not large. Due to the remote location of most tourist attractions and weak food supervision capabilities, small workshops and self-employed individuals are the main forces in the production and operation of tourist food. These practitioners lack safety and hygiene awareness and have not received relevant food safety training. In the market competition, the strategy of sacrificing quality to reduce prices is often chosen, which brings serious hidden dangers to the food safety of tourist attractions [11–15]. These issues motivated us to devise a novel approach to evaluate food safety and quality using intelligent methods. The major contributions of this paper are as follows:

- Studying the evaluation of food safety and quality extensively.
- Designing a deep learning-based method for evaluating food safety and quality using the AMCNN method.
- Performing detailed experimentation to support the effectiveness and efficiency of the proposed system compared with existing algorithms.

The remainder of the paper is structured as follows.  Section 2 discusses the state-of-the-art works related to food safety and quality.  Section 3 shows the proposed AMCNN method. Experimental results for the evaluation of food safety and quality using AMCNN with comparative analysis are presented in Section 4.  Section 5 concludes the research work with future directions.

## 2. Related Work

Tirado et al. [16] studied the causes of food safety problems from the perspective of market information and derived the theory of information asymmetry. It is believed that because food producers and operators have more food safety information than consumers, they may conceal, distort, or mislead consumers under the drive of their interests, resulting in information asymmetry between producers and consumers in the food market. Carvalho [17] believes that information should be collected correctly to ensure accurate information, and accurate information should be shared among government agencies, scientific research institutions, food production and processing enterprises, and consumers to increase information transparency. Srey et al. [18] divided food safety and quality information into two categories; the first is incomplete and asymmetric information, and the second is incomplete but symmetric information. The government's supervision of food safety can improve the efficiency of information transmission and completeness of information. Jacxsens et al. [19] believe that regulation is the government's use of legal deterrence to restrict the free choice of individuals and organizations, and its purpose is to restrict the decision-making behavior of economic subjects.

Havelaar et al. [20] established a food safety risk analysis system covering the entire food chain, and it is one of the countries with the most complete food safety guarantee measures. These perfect laws, regulations, and specific regulations cover all food categories, and at the same time, they involve all links in the production and circulation of food safety. That is, the whole process of supervision from farmland to dining table is realized. King et al. [21] analyzed the food safety system, and the specific content includes the connection between the public and the individual food safety supervision system, various options for public food safety standards, policy methods to regulate food safety, and domestic food safety supervision methods. Ortega et al. [22] combined Rosen's competitive enterprise production quality differential product model and Waldman's quality-adjusted cost function model and proposed a food safety supervision theory closely related to benefits. Panghal et al. [23] believe that currently, countries in the world have roughly formed two different food safety supervision modes. One is a mode in which multiple ports are jointly responsible for management, and the other is a mode in which a single independent port performs unified management.

Nguyen-Viet et al. [24] conducted a systematic study of the food safety supervision systems in developed countries and clearly pointed out that the unified legislative system and law enforcement system formed in food safety in developed countries lack food safety. Kotsanopoulos and Arvanitoyannis [25] combined the relevant theories of the benefit mechanism to conduct research on the distribution of benefits among food safety-related subjects. And it analyzes how the mode of food safety regulation can realize the optimal allocation of social resources. Lu et al. [26] emphasize that relevant subjects will actively interfere with food safety in order to obtain greater economic benefits. However, the current food safety management system ignores the interest mechanism of the relevant subjects and fails to effectively coordinate the interests of the subjects. Langiano et al. [27] analyzed the processing system and effects of food safety incidents and highly affirmed the role of the food safety early warning system in the food safety assurance system and believed that the construction of the food safety guarantee system should be based on the early warning mechanism, establish corresponding mechanisms and methods, and introduce relevant professionals.

Belluco et al. [28] systematically analyzed the success of the food safety assurance system and consumer trust system and believed that the construction of the food safety assurance system had played a role in promoting the overall development of the national economy. Barlow et al. [29] affirmed the achievements in food safety testing at this stage but also pointed out the defects in this aspect and believed that improving food safety-related testing technology is the basic premise to ensure the implementation of the food safety system and that capital investment and policy guidance in relevant aspects should be increased. Feng and Sun [30] systematically analyzed the current situation and trend of the construction of food safety assurance systems. Combined with the current situation, it is proposed that the construction of the food safety guarantee system is an important aspect involving people's livelihoods, and any defect may have an impact on people's lives and health. Doyle and Glass [31] carried out a study based on the current development status of the food safety guarantee system and systematically elaborated on tourism food, food hygiene, and other aspects. They believe that the government plays an important role in food safety assurance, and the government's punishment for hidden food safety hazards is directly related to the occurrence of food safety problems. However, it cannot fundamentally prevent the occurrence of food safety and hygiene incidents. Combining government supervision, control with market behavioral norms, and the mass participation of the people is the basic premise for maximizing the function of the food safety guarantee system.  Table 1 presents the summary of the state-of-the-art approaches.

## 3. Method

This work combines the safety and quality of tourism food with neural networks and proposes an AMCNN to realize the safety and quality evaluation of tourism food.

### 3.1. Basis of Convolutional Neural Networks (CNN)

The convolutional neural network is developed from the multilayer perceptron, which overcomes the defect that the multilayer perceptron network is difficult to extract high-dimensional feature information from. The CNN method is widely adopted in several applications, such as hand-gesture recognition [32] and sign language detection [33]. The input, convolutional layer, pooling layer, fully connected layer, and output layers make up the bulk of a convolutional neural network. A nonlinear feature extraction capability is improved by adding an activation function between the convolution layer and the pooling layer, which are continually superimposed for the purpose of extracting image features. To complete the sample classification, the collected features are transferred to the fully connected layer.

The convolutional layer uses the local connection to extract local information, which is the basic unit. Each convolution layer is composed of a certain number of convolution kernels and bias items of the same size, and local perception and feature extraction are performed on image features through multiple convolution kernels. The initial part of the convolutional layer mainly extracts local information such as edges and textures, while the second half of the convolutional layer can iteratively abstract and integrate local features so as to extract global features with better discrimination. During network training, the BP is utilized to continuously adjust the parameters of the convolution unit to obtain the best extraction effect. And by changing the number, size, stride, and other convolution parameters of the convolution kernel of the convolution layer, one can get different feature maps. The convolution operation is as follows:

(1) $$\begin{array}{c} x_{j}^{m}=f\left(\sum_{j}x_{i}^{m-1}*w_{ij}^{m-1}+b_{i}^{m}\right). \end{array}$$

The pooling layer is mainly located between the two convolutional layers, and its function is to reduce the dimension of features while preserving useful information as much as possible. It can extract main features, remove irrelevant information, and reduce the parameters of the model. The pooling process is invariant to rotation, translation, scaling, and so on and reduces the size of the originally large feature map. This greatly reduces the parameters in the next layer, reduces the amount of parameter calculation, and avoids the occurrence of overfitting. Commonly used pooling layers include an average pooling layer and a maximum pooling layer. Average pooling is to select all elements in a specified rectangular area and take the average value as a new feature value. Maximum pooling is to select all elements in the specified rectangular area and take the maximum value as the new feature value. The pooling operation is as follows:

(2) $$\begin{array}{c} x_{j}^{m}=f\left(\beta \times \text{down}\left(x_{i}^{m-1}\right)+b_{j}^{m}\right). \end{array}$$

The FC layer, as the name indicates, links two neurons with weights, and the fully connected layer is often located at the end of the convolutional neural network. To extract features from the data, a convolution and pooling process are used. After that, all of the newly acquired feature information is transferred to the sample space via the completely linked layer, allowing the samples to be fully feature classified. The FC operation is as follows:

(3) $$\begin{array}{c} x_{j}^{m}=f\left(\sum_{i}x_{i}^{m-1}*w_{ij}^{m-1}+b_{i}^{m}\right). \end{array}$$

The activation function is generally used after the convolution and pooling operations, and the basic convolution modules composed of the same convolution layer and pooling layer are continuously stacked to complete the feature extraction. Among them, the convolution operation extracts features, the pooling operation completes data dimensionality reduction, and the activation function introduces nonlinear mapping. All the three are progressive. This enables the convolutional neural network to approximate any nonlinear function curve, extract complex and diverse nonlinear features, and solve complex practical problems.

(4) $$\begin{array}{c} \text{Sigmoid}\left(x\right)=\frac{1}{\left(1+e^{-x}\right)},\\ \text{Tanh}\left(x\right)=\frac{\left(e^{x}-e^{-x}\right)}{\left(e^{x}+e^{-x}\right)},\\ \text{ReLU}\left(x\right)=\max\left(0,x\right). \end{array}$$

The Sigmoid function maps the input value to a fixed interval and performs well in multiclassification problems, but the function has obvious shortcomings. First, if the input is far to the left or right of the origin, the gradient value passed will be wirelessly close to 0. This results in slow parameter updates, long network training times, and, worse, gradient explosion and gradient vanishing problems. Secondly, the function contains exponential exponentiation, which requires a large amount of computation and slow training. Finally, its mean is not 0, and the resulting gradient is always positive or negative. The center point of the Tanh function image is 0, and the output value ranges from −1 to 1. This function is very similar to the Sigmoid function, but it has a wider sensitive area and is easier to train. The function still has the problem of saturation and exponentiation, so the disappearance of the gradient is also an inevitable disadvantage of a large amount of calculation.

The ReLU function is only derivable in the positive interval, and the derivative is always 1, which effectively solves the problem of vanishing gradients in backpropagation calculations. And the function structure is very simple; the positive and negative intervals are linear functions, the calculation amount is extremely small, and the calculation speed and convergence speed are very fast. The output of the negative interval of the function is always 0, and the neurons in it will not be trained. This makes neurons more sparse, reduces the interference of irrelevant information, and helps to better extract relevant features. The disadvantage of the ReLU function is that the gradient of some neurons may always be 0, which makes the neurons inactivated, and some parameters cannot be learned.

### 3.2. Xception Structure

On the basis of Inception V3, the Xception network model integrates depthwise-separable convolution into the network model. As part of the Inception network, the convolution calculation procedure is broken up into numerous distinct processes in order to fully decouple spatial correlation and cross-channel correlation. For the Inception module, cross-channel and spatial correlations are initially addressed. The standard Xception structure is shown in Figure 1. Subsequent research removes the average pooling in the standard Inception module in Inception V3 and simplifies it to only use a 3 × 3 convolution kernel. A further refinement module uses 1 × 1 convolution to perform spatial convolution.

The higher the channel blocks, the more plausible the assumption of complete decoupling of spatial and cross-channel correlations. With the above analysis, Xception is proposed. It first maps the cross-channel correlation through a 1 × 1 convolution and then maps the spatial correlation in a separate space on the output channel of the convolution. Xception can realize that each channel corresponds to one block, making the convolution separable. In Xception, a connection structure similar to ResNet's residual structure is used, which greatly speeds up the convergence speed while using depthwise-separable convolution to increase the network width. Xception is demonstrated in Figure 2.

In the evaluation of tourism food safety quality, Xception not only reduces the number of network model parameters but also improves representation for the network and improves performance for tourism food safety quality evaluation.

### 3.3. CBAM Mechanism

From a mathematical point of view, the attention mechanism is essentially a weighted operation and the distribution of weights. For the critical and effective part of the feature information, a relatively large weight will be assigned to the part. For the feature information that is not useful, a relatively small weight is assigned. The purpose is to strengthen effective information and suppress useless information.

All CNNs may use CBAM, which is an efficient and straightforward module. The module is gradually merged into an attention map in spatial and channel dimensions in the intermediate feature map. A multiplier is used to increase the number of optimal features based on the input feature map and attention map.

The connection between feature channels is used by the channel attention module to produce a channel attention map. Each channel for the feature map is a detector, so spatial dimension is reduced to further increase computational efficiency. The most common method for aggregating spatial data is to use average pooling. More precise channel attention may be obtained using maximum pooling, which primarily extracts another unique object characteristic clue. As a result, the employment of both max and average pooling layers can greatly boost the network model's capacity to represent data. It is typically not recommended to utilize two pooling layers alone.

(5) $$\begin{array}{c} M_{c}\left(F\right)=\sigma \left(W_{1}\left(W_{0}\left(F_{GAP}^{c}\right)\right)⊕W_{1}\left(W_{0}\left(F_{GMP}^{c}\right)\right)\right),\\ F_{c}=F⊗M_{c}. \end{array}$$

The spatial attention module forms a spatial attention map based on spatial relationships. The difference from channel attention is that spatial attention focuses on location. When computing spatial attention, average pooling and max pooling are used first. These two functions are combined to form feature descriptors, and pooling operations are applied along the channel axis to make the information regions more prominent.

(6) $$\begin{array}{c} M_{s}\left(F\right)=\sigma \left(f\left(F_{GAP}^{s};F_{GMP}^{s}\right)\right),\\ F_{s}=F⊗M_{s}. \end{array}$$

CBAM mainly consists of two steps. First, in terms of channel dimension, two channel descriptors are pooled using max pooling and average pooling, and the two channel descriptors are merged by channel dimension at the same time. Second, the information is compressed into one channel descriptor using global average pooling and global max pooling in the spatial dimension of the merged channel descriptors. The weight matrix aggregated in the compression operation is calibrated, and the dependencies between pixels are modeled on the basis of the above operations. The feature map is then convolved with a hidden layer containing a single convolution kernel to generate the final weight calibration.

### 3.4. Multiscale Convolutional Unit

This research develops the Xception network model for the quality of tourism food safety by widening the receptive field and extracting crucial and richer information to improve the evaluation performance. Depth-separable convolution is the foundation of the Multiscale Convolutional Unit (MCU).  Figure 3 depicts the three depth-separable convolution modules, each with a distinct kernel and residual structure.

The MCU replaces the original single convolution kernel with 3 × 3, 5 × 5, and 7 × 7 convolution kernels, respectively. They can extract different features, and the fusion of their features can generate richer feature information, improve representation for network models, and thus improve the performance.

### 3.5. AMCNN Pipeline

The network structure of the attention-based multiscale lightweight network (AMCNN) designed in this paper is illustrated in Figure 4.

First, the data is input into two 3 × 3 convolutions with 8 channels for shallow feature extraction. Then, the features of tourism food safety and quality data are extracted by MCU. The number of channels is 16, and the step size is 2. A total of 48 output channels may be generated from the fusion of characteristics derived from separate receptive fields. This is followed by four depthwise-separable convolution modules, which extract features from the fused data and build up a multiscale Xception model. As a final step, the attention module is implanted into the final network model, which selects the most important aspects from the data and eliminates all other nonessential ones. Then, global average pooling is performed and sent to softmax for tourism food safety and quality assessment.

Machine learning and deep learning-based methods are widely used in food safety review, food processing monitoring, foreign object recognition, and other domains. These approaches offer researchers and businesses faster and more efficient working systems and make it possible for customers to acquire safer food. The systems' processing capacity can be enhanced to a large extent, especially when using machine learning or deep learning methods.

## 4. Experiment

### 4.1. Experimental Detail

This work uses a self-made dataset for related experiments, which contains a total of 29,038 training samples and 12,031 test samples. The input feature of each sample is an 8-dimensional feature, and the specific information is shown in Table 2. To accommodate the input of the CNN, it is replicated to a size of 256 × 256, and the tourism food safety quality is divided into four levels. The software and hardware environment used in the experiment is shown in Table 3, and the performance indicators are accuracy and recall.

### 4.2. Experiment on Training Loss

Firstly, the extremely important training process in the neural network is analyzed, and the change in the training error of the network is illustrated in Figure 5.

In the beginning, as the amount of training increases, the loss decreases rapidly. After reaching a certain number of iterations, the loss no longer decreases significantly, indicating that the convergence state has been reached.

### 4.3. Experiment on Method Comparison

To verify the effectiveness and advancement of the AMCNN method in this work, it is compared with other methods. The experimental results are illustrated in Table 4.

AMCNN can achieve 93.7% accuracy and 91.1% recall, corresponding to the best performance in the table. Compared with the CNN method, 1.6% accuracy improvement and 1.5% recall improvement can be obtained.

### 4.4. Experiment on Xception

To verify the effectiveness of using the Xception structure in this work, we compared it with the performance when using Inception. The rest of the parameters of the network remain the same, and the experimental results are illustrated in Figure 6.

Compared with using the traditional Inception structure, using Xception can achieve 1.8% accuracy and a 1.4% recall improvement. This verifies the validity of using the latter in this work.

### 4.5. Experiment on CBAM

To verify the effectiveness of this work using the CBAM attention mechanism, we compared it with the performance without CBAM. The rest of the experimental parameters remain unchanged, and the experimental results are illustrated in Figure 7.

Compared with not using the CBAM attention module, we can get a 2.3% accuracy improvement and a 1.8% recall improvement after using this module. This proves that CBAM can guide the network to learn more discriminative features, thereby improving model performance.

### 4.6. Experiment on MCU

To verify that the multiscale features extracted by the MCU module can promote model optimization, the performance without MCU is compared with the evaluation performance after using MCU. The experimental results are illustrated in Figure 8.

Compared with not using the MCU attention module, we can get a 2.6% accuracy improvement and a 2.4% recall improvement after using this module. This shows that multiscale features can effectively improve network performance.

### 4.7. Experiment on Activation Function

This work compares the effects of different activation functions on network performance, and the compared methods are Sigmoid, Tanh, and ReLU. The rest of the experimental parameters are set unchanged, and the experimental results are illustrated in Table 5.

Compared with the Sigmoid and Tanh activation functions, the ReLU activation function can achieve the best performance improvement. Therefore, in this work, ReLU is uniformly used for nonlinear processing of features. The proposed model can be enhanced by devising distributed neural networks, which works in a decentralized structure [34, 35]. The distributed neural networks can be trained using two methods such as parallelism and model parallelism. In data parallelism, the data is segmented into partitions, where the number of partitions is equal to the total number of nodes in the compute cluster. In model parallelism, the model is divided into various parts that can run simultaneously in different nodes, and each one will run on the same data.

## 5. Conclusion

Tourism food safety refers to various safety problems that may be caused by the food consumed by tourists in the process of tourism. It includes the main aspects of tourists eating in vehicles or scenic spots during the travel process, purchasing various local specialty foods, or picking their own food during the travel process. Due to the rapid increase of the current national income level, tourism has become the main consumption mode of people in modern society and an important part of the national economy, and the food safety associated with tourism has also attracted attention. Therefore, it becomes an important task to evaluate the safety of tourist food. This work combines it with neural networks and proposes an AMCNN to realize the safety and quality evaluation of tourist food. First, this work selects Xception as the base network. Secondly, in order to extract more abundant features of information about tourism food safety and quality, the depthwise-separable convolution in the network has improved. It uses depth-separable modules with different convolution kernels to extract data features at multiple scales and, at the same time, fuse the extracted multiscale feature information. Finally, the convolutional attention module is introduced on this basis to strengthen the effective feature information in channel and space and suppress the useless feature information. Extensive experiments verify the feasibility of the AMCNN method for food safety and quality evaluation. The proposed model can be enhanced by devising distributed neural networks, which works in a decentralized structure. The accuracy of the model can be further improved by utilizing optimization methods.

## Figures and Tables

**Figure 1:** The pipeline of Inception.

**Figure 2:** The pipeline of Xception.

**Figure 3:** The structure of MCU.

**Figure 4:** The structure of AMCNN.

**Figure 5:** The training loss of AMCNN.

**Figure 6:** Comparison of Xception and Inception.

**Figure 7:** Comparison of no CBAM and having CBAM.

**Figure 8:** Comparison of no MCU and having MCU.

**Table 1:** Summary of various existing approaches.

Approach	Author	Year	Description	Benefits	Limitations

Study on climate change and food safety	Tirado et al. [16]	2010	This work made a detailed review of the potential effects of predicted changes in climate on food adulteration and food safety at various phases of the food chain and found adaptation strategies and research focus to report food safety allegations of climate change	Authors addressed the food safety implications of climate change with the help of various adaptation strategies, predictive modeling, and monitoring	The frameworks used to analyze the impacts of climate change on food safety, variability, vulnerability, and adaptation are not discussed in detail

Development of the food safety performance analysis	Jacxsens et al. [19]	2010	This work discusses the development of food safety performance indicators (FSPI) for the purpose of obtaining a first indication of the microbiological food safety performance of an implemented food safety management system (FSMS)	This is a useful tool to acquire a first sign about the microbiological performance of an implemented FSMS	Analysis of the food safety performance diagnosis for the level of governments or sector organizations is not addressed

Study on future challenges to microbial food safety	Havelaar et al. [20]	2010	This work deliberates new challenges to food safety that are caused by microorganisms as well as approaches and methodologies to counter these challenges, such as molecular methods for complex food analysis	This work has developed new definitions which are pertaining to food safety and risk framework and discussed the trends and future developments in food safety	Experimental analysis of molecular methods for complex food analysis is not performed

Random parameters logit (RPL) and latent class model (LCM)	Ortega et al. [22]	2011	In this work, measurement of consumer preferences for selecting food safety attributes in pork and food safety risk perceptions are taken into account using RPL and LCM	With the help of RPL and LCM, heterogeneity in consumer preferences is captured	A welfare analysis of the effectiveness of several food safety substantiation mechanisms from a public health viewpoint is not addressed

Statistical analysis of food safety at home using EPIINFO 3.5 statistical program	Langiano et al. [27]	2012	This work tries to outline food safety and risk insight of food-borne diseases in the private home setup and find precise behaviors during food purchase, storage, and preparation in a study	This work test the relationship between demographic characteristics and knowledge/behaviors of food diseases	Demonstration of statistical analysis is not given, and the number of samples for the study is not large

Application of hyperspectral imaging in food safety inspection and control	Feng and Sun [30]	2012	This work offers an extensive review of the application of hyperspectral imaging in the determination of physical, chemical, and biological contamination of food products	It offers fast and nondestructive methods for sensing the safety and control situation of production using hyperspectral imaging	Wide applications of hyperspectral imaging, such as familiarizing different spectral profiles, that is, NIR, Raman, and fluorescence spectra, are not investigated

Review of formation in food industries	Srey et al. [18]	2013	This work summarizes the issues of biofilms in food industries and the present and ground-breaking control strategies that have been used to battle the challenges caused by biofilms	This work briefly discusses biofilm formation and problems in the food industry due to biofilm and biofilm control strategies	The concepts related to economic and environmentally friendly control strategies are not investigated, which are crucial to satisfy the need for industrial food safety

Review of edible insects from food safety and nutritional perspective	Belluco et al. [28]	2013	This work presents a comprehensive study on taking insects as food safety and discusses nutritional facts	This work evaluates how insects are perhaps safely used as food and deliberates nutritional data to justify why insect food sources can no longer be unkempt	The way to reduce exposure to contaminants and achieve a high-quality diet when insects are taken as food is not addressed
Study on impacts of soil and water pollution on food safety and health risks	Lu et al. [26]	2015	In this work, soil and water pollution intimidation to food safety in China is discussed, and integrated policies addressing soil and water pollution for accomplishing food safety are recommended to yield a holistic approach	This work clearly investigates the factors influencing food safety and pollutants which affect the same	Resolving the issues faced due to heavy metals for food safety is not addressed

Study on the role of hazard and risk-based approaches in ensuring food safety	Barlow et al. [29]	2015	This work discusses the pros and cons of hazard- and risk-based approaches for ensuring the safety of food chemicals, allergens, ingredients, and microorganisms	This work explores the use of hazard- and risk-based approaches and summarizes the main issues discussed at the International Life Sciences Institute (ILSI) Workshop	Detection of risks for chemicals and uncertainties in risk assessment is not investigated

Study on pesticides, environment, and food safety	Carvalho [17]	2017	This work studies the major issues linked to pesticide residues, environmental fate, and effects and deliberates pathways for improved food safety	This work discusses the role of fertilizers and pesticides in agriculture and environmental fate and the effects of pesticide residues and residues in soils and aquatic environments extensively	Alternative paths to food production, the food production with better quality, and the issues in genetically modified organisms (GMOs) are not addressed

Study on food safety for food security	King et al. [21]	2017	This study discusses how present developments and trends related to food safety will influence the food sector and ultimately the ability of the sector to bring food security	This work details food safety challenges and new demands originating from producers, manufacturers, marketers, retailers, and regulators, which are created by current worldwide trends, including climate change, a growing and aging population, and urbanization	Flexible and responsive approach to addressing food challenges such as global food security is not addressed

Perspectives on food safety in Vietnam	Nguyen-Viet et al. [24]	2017	This work elaborates on some perspectives on food safety in Vietnam from the point of view of an international research institution doing food safety with partners in the country. This work concludes that the major issue of food safety in Vietnam is that certain food value chain stakeholders lack ethics	This study investigates good experiences in food safety management from other countries and learning experiences for Vietnam on how to better deal with the current food safety situation	The standard framework and regulations for food safety are not addressed

Review of food safety management systems	Panghal et al. [23]	2018	The role of study on food safety management system (FSMS) in executing food safety throughout the food production and supply chain is reviewed in this work	This work will be beneficial to industries, technical persons, academicians, researchers, and policy framers for ensuring safe production, distribution, and consumption of food	Entire technical aspects and requirements to implement the FSMS are not discoursed upon

**Table 2:** The information of data feature.

Index	Feature

*X*_1_	Mycotoxin
*X*_2_	Industrial source pollutant
*X*_3_	Phytotoxin
*X*_4_	Unbalanced diet structure
*X*_5_	Algal toxin
*X*_6_	Microbial contamination
*X*_7_	Food additive
*X*_8_	Chemical pesticide residues

**Table 3:** The experimental platform.

Item	Name

Operating system	Ubuntu 18.04
GPU	GTX 1080Ti
Memory	32 GB
Framework	TensorFlow

**Table 4:** Result of method comparison.

Method	Accuracy	Recall

SVM	87.9	86.2
BP	90.4	87.6
CNN	92.1	89.6
AMCNN	93.7	91.1

**Table 5:** Comparison of different activation functions.

Activation function	Accuracy	Recall

Sigmoid	92.4	89.1
Tanh	93.1	89.9
ReLU	93.7	91.1

## Data Availability

The datasets used during the current study are available from the corresponding author upon reasonable request.

## References

[1] Lee Y., Pennington-Gray L., Kim J. (2019). Does location matter? Exploring the spatial patterns of food safety in a tourism destination[J]. *Tourism Management*.

[2] Tarulevicz N., Ooi C. S. (2021). Food safety and tourism in Singapore: between microbial Russian roulette and Michelin stars. *Tourism Geographies*.

[3] Ghafoor K. Z., Kong L., Zeadally S. (2020). Millimeter-wave communication for internet of vehicles: status, challenges, and perspectives[J]. *IEEE Internet of Things Journal*.

[4] Zsarnoczky M. B., Zsarnoczky-Dulhazi F., Adol G. F. C., Barczak M., David L. D (2019). Food safety challenges in the tourism processes. *Rural Sustainability Research*.

[5] Okumus B. (2020). Food tourism research: a perspective article. *Tourism Review*.

[6] Mahfud T., Pardjono D., Lastariwati B (2019). CHEF’S competency as a key element in food tourism success: a literature review. *Geo Journal of Tourism and Geosites*.

[7] Muangasame K., Park E. (2019). Food tourism, policy and sustainability: behind the popularity of Thai food[M]. *Food Tourism in Asia*.

[8] Cha J. M., Borchgrevink C. P. (2019). Customers’ perceptions in value and food safety on customer satisfaction and loyalty in restaurant environments: moderating roles of gender and restaurant types. *Journal of Quality Assurance in Hospitality & Tourism*.

[9] Kwol V. S., Avci T., Eluwole K. K., Dalhatu A (2020). Food safety knowledge and hygienic‐sanitary control: a needed company for public well‐being. *Journal of Public Affairs*.

[10] Zrnić M., Brdar I., Kilibarda N. (2021). The importance of traditional food quality — the viewpoint of the tourism. *Meat Technology*.

[11] Park E., Kim S., Yeoman I. (2019). Eating in asia: understanding food tourism and its perspectives in asia[M]. *Food Tourism in Asia*.

[12] Lee H. F., Boccalatte M. (2019). Food safety in China from North American and European perspectives. *Asian Geographer*.

[13] Kogan N. E., Bolon I., Ray N. (2019). Wet markets and food safety: TripAdvisor for improved global digital surveillance. *JMIR public health and surveillance*.

[14] Bansah A. K., Adam I., Hiamey S. E. (2021). Segments of cognitive responses towards local food safety concerns amongst international students in Ghana: segments of cognitive responses towards local food safety concerns amongst international students in Ghana[J]. *African Journal of Hospitality and Tourism Management*.

[15] Lee Y. J. A., Jang S., Kim J. (2020). Tourism clusters and peer-to-peer accommodation. *Annals of Tourism Research*.

[16] Tirado M. C., Clarke R., Jaykus L. A., McQuatters-Gollop A., Frank J (2010). Climate change and food safety: a review. *Food Research International*.

[17] Carvalho F. P. (2017). Pesticides, environment, and food safety. *Food and energy security*.

[18] Srey S., Jahid I. K., Ha S. D. (2013). Biofilm formation in food industries: a food safety concern. *Food Control*.

[19] Jacxsens L., Uyttendaele M., Devlieghere F., Rovira J., Gomez S. O., Luning P (2010). Food safety performance indicators to benchmark food safety output of food safety management systems. *International Journal of Food Microbiology*.

[20] Havelaar A. H., Brul S., De Jong A., de Jonge R., Zwietering M. H., ter Kuile B. H (2010). Future challenges to microbial food safety. *International Journal of Food Microbiology*.

[21] King T., Cole M., Farber J. M. (2017). Food safety for food security: r. *Trends in Food Science & Technology*.

[22] Ortega D. L., Wang H. H., Wu L., Olynk N. J (2011). Modeling heterogeneity in consumer preferences for select food safety attributes in China. *Food Policy*.

[23] Panghal A., Chhikara N., Sindhu N., Jaglan S (2018). Role of food safety management systems in safe food production: a review. *Journal of Food Safety*.

[24] Nguyen-Viet H., Tuyet-Hanh T. T., Unger F. (2017). Food safety in Vietnam: where we are at and what we can learn from international experiences[J]. *Infectious diseases of poverty*.

[25] Kotsanopoulos K. V., Arvanitoyannis I. S. (2017). The role of auditing, food safety, and food quality standards in the food industry: a review. *Comprehensive Reviews in Food Science and Food Safety*.

[26] Lu Y., Song S., Wang R. (2015). Impacts of soil and water pollution on food safety and health risks in China. *Environment International*.

[27] Langiano E., Ferrara M., Lanni L., Viscardi V., Abbatecola A. M., De Vito E (2012). Food safety at home: knowledge and practices of consumers. *Journal of Public Health*.

[28] Belluco S., Losasso C., Maggioletti M., Alonzi C. C., Paoletti M. G., Ricci A (2013). Edible insects in a food safety and nutritional perspective: a critical review. *Comprehensive Reviews in Food Science and Food Safety*.

[29] Barlow S. M., Boobis A. R., Bridges J. (2015). The role of hazard- and risk-based approaches in ensuring food safety. *Trends in Food Science & Technology*.

[30] Feng Y. Z., Sun D. W. (2012). Application of hyperspectral imaging in food safety inspection and control: a review. *Critical Reviews in Food Science and Nutrition*.

[31] Doyle M. E., Glass K. A. (2010). Sodium reduction and its effect on food safety, food quality, and human health. *Comprehensive Reviews in Food Science and Food Safety*.

[32] Gadekallu T. R., Alazab M., Kaluri R. (2021). Hand gesture classification using a novel CNN-crow search algorithm[J]. Complex and Intelligence System.

[33] Mannan A., Abbasi A., Javed A. R., Ahsan A., Gadekallu T. R., Xin Q (2022). Hypertuned deep convolutional neural network for sign language recognition. *Computational Intelligence and Neuroscience*.

[34] Kumar R., Tripathi R. (2020). Secure healthcare framework using blockchain and public key cryptography[C]. *Blockchain Cybersecurity, Trust and Privacy*.

[35] Kumar R., Tripathi R. (2021). DBTP2SF: a deep blockchain‐based trustworthy privacy‐preserving secured framework in industrial internet of things systems. *Transactions on Emerging Telecommunications Technologies*.

